The article "Effects of Knee Flexion Angles on the Joint Force and Muscle Force during Bridging Exercise: A Musculoskeletal Model Simulation" was published in 2022. Journal: J Healthc Eng.

# Effects of Knee Flexion Angles on the Joint Force and Muscle Force during Bridging Exercise: A Musculoskeletal Model Simulation

**DOI:** 10.1155/2022/7975827

**Published:** 2022-05-29

**Authors:** Yasufumi Takeshita, Masayuki Kawada, Takasuke Miyazaki, Yuki Nakai, Sota Araki, Shintaro Nakatsuji, Yuta Matsuzawa, Shobu Nakashima, Ryoji Kiyama

**Affiliations:** ^1^Doctoral Program, Course of Health Sciences, Graduate School of Health Sciences, Kagoshima University, 8-35-1 Sakuragaoka, Kagoshima City, Kagoshima 890-8544, Japan; ^2^Department of Physical Therapy, School of Health Sciences, Faculty of Medicine, Kagoshima University, 8-35-1 Sakuragaoka, Kagoshima City, Kagoshima 890-8544, Japan; ^3^Department of Orthopaedic Surgery, Graduate School of Medical and Dental Sciences, Kagoshima University, 8-35-1 Sakuragaoka, Kagoshima City, Kagoshima 890-8520, Japan; ^4^Department of Mechanical Systems Engineering, Faculty of Engineering, Daiichi Institute of Technology, 1-10-2 Kokubuchuoh, Kirishima City, Kagoshima 899-4395, Japan; ^5^Miyakonojo Rehabilitation Academy, 5822-9 Oiwadacho, Miyakonojo City, Miyazaki 885-0062, Japan; ^6^Master's Program, Course of Health Sciences, Graduate School of Health Sciences, Kagoshima University, 8-35-1 Sakuragaoka, Kagoshima City, Kagoshima 890-8544, Japan

## Abstract

Bridging exercise is commonly used to increase the strength of the hip extensor and trunk muscles in physical therapy practice. However, the effect of lower limb positioning on the joint and muscle forces during the bridging exercise has not been analyzed. The purpose of this study was to use a musculoskeletal model simulation to examine joint and muscle forces during bridging at three different knee joint angle positions. Fifteen healthy young males (average age: 23.5 ± 2.2 years) participated in this study. Muscle and joint forces of the lumbar spine and hip joint during the bridging exercise were estimated at knee flexion angles of 60°, 90°, and 120° utilizing motion capture data. The lumbar joint force and erector spinae muscle force decreased significantly as the angle of the knee joint increased. The resultant joint forces were 200.0 ± 23.2% of body weight (%BW), 174.6 ± 18.6% BW, and 150.5 ± 15.8% BW at 60°, 90°, and 120° knee flexion angles, respectively. On the other hand, the hip joint force, muscle force of the gluteus maxims, and adductor magnus tended to increase as the angle of the knee joint increased. The resultant joint forces were 274.4 ± 63.7% BW, 303.9 ± 85.8% BW, and 341.1 ± 85.7% BW at a knee flexion angle of 60°, 90°, and 120°, respectively. The muscle force of the biceps femoris decreased significantly with increased knee flexion during the bridging exercise. In conclusion, the knee flexion position during bridging exercise has different effects on the joint and muscle forces around the hip joint and lumbar spine. These findings would help clinicians prescribe an effective bridging exercise that includes optimal lower limb positioning for patients who require training of back and hip extensor muscles.

The article "Effects of Knee Flexion Angles on the Joint Force and Muscle Force during Bridging Exercise: A Musculoskeletal Model Simulation" was published in 2022. Journal: J Healthc Eng.

## 1. Introduction

Optimal hip extensor and trunk muscle strength have been associated with injury prevention, pain reduction, and an enhancement of athletic performance [1–4]. Bridging exercise is an accepted component of physical therapy programs that assist in strengthening these muscle groups of the back. Muscle activity during the bridging exercise has been analyzed with electromyography (EMG) [5–8]. These studies revealed that the activities of the biceps femoris and erector spinae are greater during bridging than during walking. However, muscle activity during the bridging exercise changes depending on the knee flexion position due to the alteration of the relative position of the joint center and the floor reaction force acting on the feet. Previous studies have focused on the muscle activity induced during various bridging exercises; however, studies examining the joint forces during bridging exercises are scarce. An increase in muscle activity during exercise is associated with increased muscle force. Previously, it has been shown that approximately 80% of the joint force depends on the tensile force generated by the muscles crossing the joint and that the contribution of muscle force towards joint force is greater than that of the ground reaction force [9]. Consequently, the knee flexion angle during bridging might affect both muscle and joint forces [10–13]. Mechanical loading has been identified as an important risk factor in the development of joint pain [14, 15]. Therefore, an understanding of joint forces during the bridging exercise could be an important factor for consideration when prescribing an appropriate physical therapy program.

Numerous studies have investigated the joint and muscle forces during static standing, gait, squatting, forward lunging, and lifting [16–18]. Joint and muscle forces were typically estimated using musculoskeletal model simulation from the kinematic and kinetic data measured by a motion capture system and a force platform. Conversely, few studies have analyzed the joint and muscle forces during supine exercise due to the difficulties of measuring the floor reaction force and analyzing the subsequent kinetic data. However, an optimization method has recently been used for estimating the floor reaction force. This method enables the estimation of the external force acting on humans so as to the external force is balanced with the gravity and the acceleration of the center of mass. This allows the kinetic analysis using a musculoskeletal model simulation in various exercises, including supine exercise, without requiring the measurement of the floor reaction force [19–21].

The article "Effects of Knee Flexion Angles on the Joint Force and Muscle Force during Bridging Exercise: A Musculoskeletal Model Simulation" was published in 2022. Journal: J Healthc Eng.

Despite the frequent utilization of the bridging exercise in physical therapy practice, the effect of lower limb position on the joint and muscle forces during bridging has largely been overlooked. The purpose of this study was to use a musculoskeletal model simulation to examine the joint and muscle forces around the hip joint and the lumbar spine during the bridging exercise performed at three knee joint angle positions. We hypothesized that the joint force in the lumbar spine and the hip decreases during bridging exercise with an increased knee flexion angle due to an decrease in the moment arm of a floor reaction force acting on the feet and around the lumbar spine and hip joint.

## 2. Materials and Methods

### 2.1. Participants

Fifteen healthy young males, with no history of neurological, respiratory, back, or lower limb pathology (age: 23.5 ± 2.2 years; height: 1.70 ± 0.1 m; weight: 61.6 ± 8.1 kg) participated in this simulation study. This study was limited to only male participants because the musculoskeletal model (AMMR, v.2.1.1, AnyBody Technology, Aalborg, DK) used in this study was based on average male characteristics. All participants provided signed informed consent. This study was approved by the Ethics Committee on Epidemiological and Related Studies at the Sakuragaoka campus of the Kagoshima University (approval number: 180113Epi ver. 2). The study was performed between June and August 2021 at the Faculty of Medicine at Kagoshima University.

### 2.2. Exercise and Motion Capture

The bridging exercise with knee flexion angles of 60°, 90°, and 120° was evaluated using a motion capture system and surface EMG. The knee flexion angles were measured using a goniometer to standardize the foot positions for the bridging exercises (Figure 1). To maximize stability, participants performed all the bridging exercises with bare feet while arms and other body parts rested on the floor. Each participant steadily raised his pelvis to his maximum hip extension angle for two seconds, held this position for one second, and lowered it for two seconds. Bridging exercises with three lower limb positions were randomly performed five times.

Motion capture was performed using an 8-camera OptiTrack Flex13 system (NaturalPoint, Corvallis, OR, USA) with a sampling frequency of 100 Hz. The validity of this system has been confirmed in previous studies [22–24]. Each subject wore 40 reflective markers based on a plug-in-gait marker set [18]. Posterior markers could not be captured in the supine posture; therefore, they were attached anteriorly to the same segment to enable capturing and defining of the local coordinate system of the segment.

The article "Effects of Knee Flexion Angles on the Joint Force and Muscle Force during Bridging Exercise: A Musculoskeletal Model Simulation" was published in 2022. Journal: J Healthc Eng.

### 2.3. Musculoskeletal Model

The present study utilized a 42 degrees-of-freedom full-body musculoskeletal model (AMMR v.2.1.1, AnyBody 7.1) for the analysis of joint and muscle forces. Marker trajectories were filtered using a Butterworth low-pass filter at a 6 Hz cut-off frequency [25]. Anthropometric data, including weight, height, and segment length, were used to scale the musculoskeletal model to match each study participant.

To estimate the external force exerted from the floor during exercise, 83 contact points between the body surface and the floor were defined on each body segment in the original model. In the supine model, one contact point was determined for the occiput, 42 points for the spine, six points for the bilateral upper limbs, eight points for the ischium, 14 points for the bilateral thighs, six points for the bilateral lower limbs, and six points for both soles (Figure 2). Contact was determined by the distance between the floor and the contact point on the body [20], and contact elements provided compressive reaction forces. The external force during bridging was estimated using an optimization algorithm to balance the motion of the human body model.

Each muscle was simulated using a three-element muscle model, consisting of a Hill-type contractile element, a parallel-elastic element, and a series-elastic element. The contractile element included the force-length and force-velocity relationships as well as the effects of the pennation angle. The parallel-elastic element consisted of a nonlinear spring whose stiffness was governed by the passive force-length relationship to the muscle. Muscle forces were computed through inverse dynamic and optimization analysis by minimizing the sum of the cubes of muscle recruitment [26, 27]. The intersegmental resultant, proximal-distal, anterior-posterior, and mediolateral joint forces acting on the lumbar (L4–L5) spinal joint and hip joint were analyzed during bridging. The joint force was calculated based on the net joint and tensile forces of the muscles crossing those joints and resolved into three components based on the reference frame of the child segment. Vertical, anterior, and medial forces were represented as positive values. The following five muscles were analyzed: gluteus maximus (GMAX), adductor magnus (ADDM), biceps femoris long head (BFLH), erector spinae (ES), and multifidus (MF). Joint and muscle forces were normalized to each participant's body weight (%BW).

The article "Effects of Knee Flexion Angles on the Joint Force and Muscle Force during Bridging Exercise: A Musculoskeletal Model Simulation" was published in 2022. Journal: J Healthc Eng.

### 2.4. Electromyography

A signal acquisition system (biosignals plux, PLUX S.A., Lisbon, Portugal) was used to measure EMG [28] based on the SENIAM (surface EMG for noninvasive assessment of muscles) recommendations [29]. The acquisition procedure followed the directives of the International Society of Electrophysiology and Kinesiology (acquisition at a sampling frequency of 1000 Hz and filtering using a band-pass filter between 10 and 500 Hz). Participants were required to undergo maximum voluntary contraction (MVC) tests for normalization. The activation of GMAX, BFLH, ES, and MF was expressed as %MVC. The normalization tests were performed based on Kendall's manual muscle testing [30]. The MVC for the GMAX was measured by the hip extension with 90° knee flexion, against the resistance applied just above the popliteal fossa in the prone position. The MVC of BFLH was measured at the 50° knee flexion, against the resistance applied just above the ankle, in the prone position. The MVC of ES and MF was measured by the trunk extension in the prone position, against the resistance applied to the upper back.

### 2.5. Statistical Analysis

The mean joint force, muscle force, and EMG data during the one-second holding position with maximum hip extension were calculated. The mean from the five trials in each bridging exercise was analyzed. The normality of distribution was tested using the Shapiro–Wilk test. If normality of distribution could be assumed, data were analyzed using the one-way repeated measures ANOVA with Schaffer's post hoc test to determine the effect of knee position during bridging exercise on joint and muscle load. If the normality of distribution could not be assumed, data were analyzed using the Friedman test with the Wilcoxon signed-rank test adjusted with the Holm post hoc test. In addition, effect sizes were expressed as *η*^2^ (0.01 = small effect, 0.06 = medium effect, and 0.14 = large effect) [31].

All statistical tests were performed using the *R* software package (version 2.8.1). For all analyses, the threshold of significance was established at an alpha of 0.05. The joint and muscle forces and EMG data determined in this study are presented as mean and standard deviations.

## 3. Results

### 3.1. Joint Force

The resultant lumbar joint force significantly decreased as the angle of knee flexion increased (*F* = 234.62, *P* < 001, *η*^2^ = 0.536) (Table 1). The resultant joint forces were 200.0 ± 23.2%BW, 174.6 ± 18.6%BW, and 150.5 ± 15.8%BW at the knee flexion angles of 60°, 90°, and 120°, respectively. The proximal-distal force was the largest, followed by the anterior force; both forces, similar to the resultant force, decreased with increasing knee flexion angle. The mediolateral force was small and did not change significantly with changes in knee flexion angle.

The article "Effects of Knee Flexion Angles on the Joint Force and Muscle Force during Bridging Exercise: A Musculoskeletal Model Simulation" was published in 2022. Journal: J Healthc Eng.

The resultant hip joint force increased as the angle of knee flexion increased (*χ*^2^ = 9.73, *P* = .008, *η*^2^ = 0.324). The resultant joint forces were 274.4 ± 63.7%BW, 303.9 ± 85.8%BW, and 341.1 ± 85.7%BW at the knee flexion angles of 60°, 90°, and 120°, respectively. The proximal-distal force was the largest of the component forces, and similar to the resultant force, it increased as the angle of knee flexion increased.

### 3.2. Muscle Forces and Electromyography

The GMAX and ADDM muscle forces increased significantly as the angle of knee flexion increased (Table 2). Conversely, the muscle forces of the MF, ES, and BFLH decreased significantly as the angle of knee flexion increased.

The MF, ES, and BFLH muscle activity decreased significantly as the angle of knee flexion increased, similar to the muscle force. In contrast, the muscle activity of the GMAX was not affected by the angle of the knee joint (Table 3).

## 4. Discussion

We analyzed the effect of knee joint angles on joint and muscle forces in the lumbar spine and the hip joint during the bridging exercise. We hypothesized that the joint forces would decrease as the knee flexion increased. Our results showed that although the lumbar joint force decreased in bridging with increased knee flexion, the hip joint did not.

The resultant lumbar joint force decreased in the bridging exercise with increased knee flexion. Similarly, the proximal, distal, and anterior lumbar forces decreased during bridging with increased knee flexion. Lumbar joint force is largely affected by ES and MF muscle forces. During bridging exercise, the external flexion moments in the lumbar and hip joints are caused by the floor reaction force acting on the bilateral feet. Thus, increasing the knee flexion angle during bridging exercise decreased the distance between the floor reaction force and the center of the lumbar and hip joints, resulting in decreased external flexion moment [9]. The observed decrease in the muscle force in the ES and MF during the bridging exercise with increased knee flexion reflects the decrease in the external lumbar flexion moment. These results are consistent with ES and MF muscle activation as measured using EMG in both the present as well as previous studies [13, 32]. Therefore, an increased knee flexion angle decreased the load on the lumbar joints and musculature during bridging exercise. Lumbar joint force during bridging ranged from approximately 150%BW to 200%BW and was larger than the previously reported joint force of 100–130%BW during walking [33, 34]. This observation suggests that although bridging is performed in a supine position, this exercise exerts a larger force on the lumbar spine than the force exerted by walking. Furthermore, these findings suggest that the physical therapists should carefully position the lower limb during bridging in order to mitigate the load on the lumbar joints and surrounding musculature.

The article "Effects of Knee Flexion Angles on the Joint Force and Muscle Force during Bridging Exercise: A Musculoskeletal Model Simulation" was published in 2022. Journal: J Healthc Eng.

Conversely, the resultant force of the hip joint increased during bridging with increased knee flexion. Similarly, proximal-distal, medial, and posterior forces increased during the bridging exercise with increased knee flexion. The hip joint force was greatly affected by the muscle force of the hip extensor muscles. The ADDM muscle force was 75.7%BW at 120° knee flexion, which was the highest among the muscles analyzed in this study. The hip extension moment is generated sequentially by the GMAX, hamstrings, and ADDM, as they cross the posterior hip joint. An increase in the knee flexion angle shortens the biceps femoris [35] and decreases the maximal force generated by the biceps femoris according to the length-tension curve. The force of the ADDM, rather than that of the hamstrings, generated the hip extensor moment as noted by increased tension force during bridging with increased knee flexion. Previous studies have reported that the moment arm of the ADDM is smaller than that of the other hip extensor muscle groups, such as the hamstrings, at a neutral hip position [36, 37]. The muscle with a short moment arm with respect to the joint center requires a larger tension force when compared to a similar joint moment generated by the muscle with a larger moment arm. Thus, the recruitment of the ADDM during bridging with increased knee flexion would increase the resultant force acting on the hip joint. Considering the pathway of this muscle, increased activation of the ADDM would also contribute to the increase in both medial and posterior forces. The largest hip joint force during bridging exercise was 341.1%BW in this study. This force is almost equivalent to that observed during walking (367–430%BW) [38, 39]. While the bridging exercise with a 120° knee flexion position is considered a supine exercise supported bilaterally by the feet and the back, a therapist should pay attention to the hip joint force.

Increased muscle force of the GMAX would also contribute to the increase in the hip joint force during bridging with increased knee flexion. However, consistent with previous studies [8, 24], GMAX activity measured using EMG during the bridging exercise was not significantly affected by the knee flexion position. The EMG muscle activity measurement is impacted by the thickness of the subcutaneous fat [40, 41], and this might be a potential factor responsible for the observed discrepancy between the GMAX muscle force estimated by the musculoskeletal simulation and the GMAX muscle activation measured using EMG.

The article "Effects of Knee Flexion Angles on the Joint Force and Muscle Force during Bridging Exercise: A Musculoskeletal Model Simulation" was published in 2022. Journal: J Healthc Eng.

This study had several limitations. Due to the difficulty of measurement in the supine position, we analyzed muscle and joint forces using floor reaction force estimated by the optimization technique. We also used surface EMG to estimate muscle activity during the bridging exercise. Although the muscle force and muscle activity were consistent in the MF, ES, and BFLH depending on the exercise conditions, the GMAX force and activity measurements were inconsistent. Also, the ADDM was not analyzed by EMG due to crosstalk. We estimated the muscle and joint forces in healthy young males by simulation using a scaled musculoskeletal model base on average male characteristics. Therefore, these results should be cautiously adapted to females, older people, and people with pathological conditions. Additional studies are required to address these issues and to perform a comprehensive analysis of the effect of the lower limb position on the muscle and joint forces around the hip joint and lumbar spine during the bridging exercise. Further investigations will also be needed to generalize these findings to people requiring exercise, including frail older people and people with lower back pain.

## 5. Conclusions

In conclusion, knee flexion during the bridging exercise has different effects on the joint forces of the lumbar spine and hip joint. Moreover, depending on the knee joint flexion position, those joint forces could be equal to or greater than those during gait. This study has provided the basic data to help clinicians prescribe the optimal lower limb position during the bridging exercise for patients who require training of the back and hip extensor muscles.

## Figures and Tables

**Figure 1:** Bridging exercises with (a) 60°, (b) 90°, and (c) 120° knee flexion positions.

**Figure 2:** Floor reaction forces during the bridging exercise estimated using the optimization technique. Floor reaction forces were estimated as the external force (blue lines) acting on the 83 contact points between the human body and the floor (green circles) using the optimization method. Contact was determined by the distance between the floor and the contact points on the body, and the sum of all predicted reaction forces balanced the sum of gravity and mass-acceleration products of all body segments.

**Table 1:** Joint forces acting on the lumbar spine and the hip joint determined using the musculoskeletal model.

Joint force (%BW)		60°	90°	120°	*χ* ^2^, F	*P*	*η* ^2^
Lumbar	Resultant	200.0 ± 23.2^*∗∗*^ ††	174.6 ± 18.6††	150.5 ± 15.8	*F* = 234.62	<0.001	0.536
	PD	141.4 ± 16.4^*∗∗*^ ††	123.4 ± 13.2††	106.4 ± 11.2	*F* = 234.57	<0.001	0.536
	AP	13.2 ± 1.3^*∗∗*^ ††	12.2 ± 1.2††	10.7 ± 1.0	*F* = 94.67	<0.001	0.462
	ML	−0.38 ± 0.91	−0.29 ± 0.65	−0.23 ± 0.52	*F* = 0.85	.407	0.008

Hip	Resultant	274.4 ± 63.7†	303.9 ± 85.8†	341.1 ± 85.7	*χ* ^*2*^ *=* 9.73	.008	0.324
	PD	192.9 ± 45.1†	213.5 ± 60.9	239.5 ± 61.0	*χ* ^*2*^ = 9.73	<0.001	0.324
	AP	−11.3 ± 6.5^*∗∗*^ ††	−17.0 ± 7.3††	−21.9 ± 8.4	*F* = 41.69	<0.001	0.268
	ML	28.7 ± 6.8^*∗∗*^ ††	33.0 ± 4.8††	38.9 ± 5.0	*F* = 38.87	<0.001	0.373

*Note*. Lumbar, L4–L5 joint force; Hip, hip joint force; Resultant, resultant force; PD, proximal distal force; AP, anterior posterior force; ML, mediolateral force; ^*∗*^*P* < 0.05 vs 90°; ^*∗∗*^*P* < 0.01 vs 90°; †*P* < 0.05 vs 120°; ††*P* < 0.01 vs 120°. Variables excluding the resultant and PD force of the hip joint were assumed to be normally distributed.

The article "Effects of Knee Flexion Angles on the Joint Force and Muscle Force during Bridging Exercise: A Musculoskeletal Model Simulation" was published in 2022. Journal: J Healthc Eng.

**Table 2:** Muscle forces determined using the musculoskeletal model.

Muscle force (%BW)	60°	90°	120°	F	*P*	*η* ^2^
Gluteus maximus	8.3 ± 8.0^*∗∗*^ ††	22.6 ± 7.6††	34.4 ± 9.8	*F* = 84.80	<0.001	0.629
Multifidus	11.3 ± 3.2^*∗∗*^ ††	9.2 ± 2.9††	7.4 ± 2.4	*F* = 103.86	<0.001	0.253
Erector supine	48.8 ± 12.5^*∗∗*^ ††	41.0 ± 11.0††	33.6 ± 9.6	*F* = 149.28	<0.001	0.252
Biceps femoris	44.8 ± 10.7^*∗∗*^ ††	21.3 ± 5.8††	3.6 ± 1.3	*F* = 208.78	<0.001	0.858
Adductor magnus	42.1 ± 15.1^*∗∗*^ ††	56.2 ± 23.4††	75.7 ± 27.1	*F* = 33.08	<0.001	0.263

*Note*. ^*∗*^*P* < 0.05 vs 90°; ^*∗∗*^*P* < 0.01 vs 90°; †*P* < 0.05 vs 120°; ††*P* < 0.01 vs 120°. All variables were assumed to be normally distributed.

**Table 3:** Muscle activity determined using electromyography.

EMG (%MVC)	60°	90°	120°	*χ* ^2^, F	*P*	*η* ^2^
Gluteus maximus	14.5 ± 8.3	16.0 ± 7.8	16.1 ± 11.8	*χ* ^*2*^ = 0.93	.627	0.031
Multifidus	40.7 ± 16.6^*∗*^ ††	36.0 ± 17.5†	31.3 ± 14.9	*F* = 9.30	< .001	0.056
Erector supine	34.4 ± 15.0^*∗∗*^ ††	27.2 ± 13.6	22.9 ± 12.7	*F* = 12.96	< .001	0.113
Biceps femoris	43.7 ± 19.6^*∗∗*^ ††	24.9 ± 14.6††	11.0 ± 11.9	*χ* ^*2*^ = 26.53	< .001	0.884

*Note*. ^*∗*^*P* < 0.05 vs 90°; ^*∗∗*^*P* < 0.01 vs 90°; †*P* < 0.05 vs 120°; ††*P* < 0.01 vs 120°. Multifidus and erector supine muscle activities were assumed to be normally distributed.

## Data Availability

The data used to support the finding of the current study are available from the corresponding author upon request.
